This article has been retracted.

# Artificial Intelligence Algorithm-Based Computerized Tomography Image Features Combined with Serum Tumor Markers for Diagnosis of Pancreatic Cancer

**DOI:** 10.1155/2022/8979404

**Published:** 2022-03-02

**Authors:** Zhengmei Qiao, Junli Ge, Wenping He, Xinye Xu, Jianxin He

**Affiliations:** ^1^Department of Clinical Laboratory, Baoji Hi-Tech Hospital, Baoji, 721013 Shaanxi, China; ^2^Liver and Gallbladder Surgery, Ankang Hospital of Traditional Chinese Medicine, Ankang, 725000 Shaanxi, China; ^3^Emergency Surgery, Ankang Hospital of Traditional Chinese Medicine, Ankang, 725000 Shaanxi, China

## Abstract

The objective of this study was to analyze the value of artificial intelligence algorithm-based computerized tomography (CT) image combined with serum tumor markers for diagnoses of pancreatic cancer. In the study, 68 hospitalized patients with pancreatic cancer were selected as the experimental group, and 68 hospitalized patients with chronic pancreatitis were selected as the control group, all underwent CT imaging. An image segmentation algorithm on account of two-dimensional (2D)-three-dimensional (3D) convolution neural network (CNN) was proposed. It also introduced full convolutional network (FCN) and UNet network algorithm. The diagnostic performance of CT, serum carbohydrate antigen-50 (CA-50), serum carbohydrate antigen-199 (CA-199), serum carbohydrate antigen-242 (CA-242), combined detection of tumor markers, and CT-combined tumor marker testing (CT-STUM) for pancreatic cancer were compared and analyzed. The results showed that the average Dice coefficient of 2D-3D training was 84.27%, which was higher than that of 2D and 3D CNNs. During the test, the maximum and average Dice coefficient of the 2D-3D CNN algorithm was 90.75% and 84.32%, respectively, which were higher than the other two algorithms, and the differences were statistically significant (*P* < 0.05). The penetration ratio of pancreatic duct in the experimental group was lower than that in the control group, the rest were higher than that in the control group, and the differences were statistically significant (*P* < 0.05). CA-50, CA-199, and CA-242 in the experimental group were 141.72 U/mL, 1548.24 U/mL, and 83.65 U/mL, respectively, which were higher than those in the control group, and the differences were statistically significant (*P* < 0.05). The sensitivity, specificity, positive predictive value, and authenticity of combined detection of serum tumor markers were higher than those of CA-50, CA-199, and CA-242, and the differences were statistically significant (*P* < 0.05). The results showed that the proposed algorithm 2D-3D CNN had good stability and image segmentation performance. CT-STUM had high sensitivity and specificity in diagnoses of pancreatic cancer.

## 1. Introduction

Pancreatic cancer is one of the malignant tumors of the digestive system. It has a high degree of malignancy, high morbidity and mortality, and poor prognosis [1, 2]. It was reported that the global incidence rate of pancreatic cancer has risen to the fourth malignant tumor after lung cancer and breast cancer. In China, the death rate of pancreatic cancer has risen in recent years [3, 4]. Surgical resection is currently the main treatment for pancreatic cancer patients; although, it can improve the survival rate of patients with pancreatic cancer. Clinical studies have reported that 85% of patients have advanced cancer at the time of hospital visit [5, 6]. Less than 20% of these patients are treated surgically, the 5-year survival rate is less than 5% on average. This is because of the rapid development of pancreatic cancer. Once the clinical symptoms appear and treatments are not timely, the average survival time of patients is less than 4 months, which seriously harms people's physical and mental health [7–9].

Clinical diagnoses of pancreatic cancer mainly depend on image examinations and serum tumor marker examinations. Image examinations include ultrasound scanning, computed tomography (CT), magnetic resonance imaging, and endoscopic examination. Among them, CT images have a relatively high resolution and do little harm to the human body and are of certain value in early diagnoses of pancreatic cancer; so, they are widely used in clinical practice [10]. However, doctors' judgments and analyses of patient images are greatly influenced by their subjective factors. The same image is judged and analyzed by different doctors. The results are affected by doctors' clinical experience and mental state at that time and are also different and time-consuming [11]. The use of serum tumor markers in the diagnosis of pancreatic cancer is also the focus of clinical research. Fujimoto et al. [12] combined the serum marker CA19-9 and methylated short stature-related transcription factor 3 (RUNX 3) in early pancreatic cancer screening and found that the sensitivity and the specificity of the two combined detection of pancreatic cancer were 85.5% and 93.5%, respectively, showing good diagnostic effect. Dong et al. [13] analyzed the diagnostic value of CA19-9, CA 242, and serum peripherin (POSTN) for pancreatic cancer and finally found that CA19-9 and CA 242 combined with POSTN detection was a potential serum marker for the diagnosis of early pancreatic cancer. Therefore, it is of great significance to assist doctors to make rapid and efficient diagnoses of the disease so that patients can receive timely and effective treatments.

In recent years, with the continuous development and improvement of artificial intelligence, some scholars have proposed to use computer aided diagnosis (CAD) to help clinicians diagnose diseases [14]. The principle of CAD is to use the intelligent computer system to automatically analyze and process patients' images, determine the lesion position in patients, and analyze the lesion situation, so as to achieve the objective of assisting doctors in diagnoses and treatments [15, 16]. Among many algorithms, deep learning technology is particularly superior to image processing. Therefore, this study considered the use of CT image features on account of the two-dimensional (2D)-three-dimensional (3D) convolution neural network (CNN) algorithm combined with serum tumor markers in clinical diagnoses of pancreatic cancer.

To sum up, it is of great significance to explore how to enable auxiliary doctors to diagnose pancreatic cancer, improve the diagnostic accuracy, and enable patients to receive timely treatments. However, 2D-3D CNN has a better segmentation effect in CT images. Therefore, this study proposed a CT image feature diagnosis model on account of the artificial intelligence algorithm, which was 2D-3D CNN. Compared with full convolutional network (FCN) and UNet algorithms, serum carbohydrate antigen-50 (CA-50), serum carbohydrate antigen-199 (CA-199), and serum carbohydrate antigen-242 (CA-242) were combined for diagnostic analyses of pancreatic cancer patients. The diagnostic performance of different detection methods was compared. The use value of CT imaging features combined with serum tumor markers on account of 2D-3D CNN in clinical diagnoses of pancreatic cancer was comprehensively evaluated, so as to provide reliable basis for diagnoses and treatments of pancreatic cancer patients.

## 2. Materials and Methods

### 2.1. Research Objects

In this study, 136 patients with pancreatic cancer or chronic pancreatitis who were in hospital from May 2017 to June 2019 were selected as the research objects. Among them, 68 patients with pancreatic cancer were used as the experimental group, and 68 patients with chronic pancreatitis were selected as the control group. The patients in the experimental group ranged in age from 37 to 76 years old, with an average age of 53.32 ± 12.57 years old, including 47 males and 21 females. In the control group, patients with chronic pancreatitis ranged from 35 to 77 years old, with an average age of 53.27 ± 11.68 years old, including 48 males and 20 females. There were no statistical differences in age, gender, and other general information between two groups (*P* > 0.05). This study has been approved by ethics committee of hospital. All the patients and their families were aware of this study and signed informed consents.

Inclusion criteria were as follows: first, pancreatic cancer and chronic pancreatitis were confirmed by pathological examinations. Second, patients were younger than 76 years old. Third, radiotherapy and chemotherapy were not performed before CT examinations. Fourth, patients' clinical data were complete.

Exclusion criteria were as follows: first, CT image quality was poor. Second, there were other systemic malignancies. Third, pregnant women and patients could not cooperate with the test.

### 2.2. CT Scan

64-slice spiral CT was used to routinely scan the upper abdomen of the patient with pancreatic cancer. The patient was instructed to maintain an empty stomach before the scan, and 500 mL of pure water was taken orally to fill the gastrointestinal tract 30 minutes before the scan. Scanning parameter setting was as the following: thickness was 3 mm, collimation was 2.5 mm, space was 1 mm, power was 120 kV, 200 mAs, and 0.5 s, and matrix reconstruction was 512 × 512. All patients received plain and 3-phase enhanced scan of upper and middle abdomen, and each scan time was 6 ~ 8 seconds. The delay time was set to 23 seconds for the arterial phase, 60 seconds for the portal pulse phase, and 40 seconds for the pancreatic phase. The contrast agent was 300 mg/mL and 90~100 mL of iodihyalcohol injection, which was injected through the forearm vein mass at a rate of 3.0 mL/s.

### 2.3. Serum Tumor Marker Test

The researchers were arranged to collect 5 mL of venous blood samples from the experimental group and control group in fasting state and put them into anticoagulant tubes containing anticoagulants. After 30 min at room temperature, the upper serum was collected by centrifugation at 4000 r/min for 5 min. The contents of CA-50, CA-242, and CA-l99 tumor markers in serum were detected strictly in line with the operation and use instructions of the kit. The positive value ranges of CA-50, CA-242, and CA-l99 were >20 U/mL, > 20 U/mL, and> 35 U/mL, respectively.

### 2.4. Design of the 2D-3D CNN Segmentation Algorithm

The automatic segmentation algorithm on account of CNN was divided into 2D and 3D methods. The 2D method took a single slice as input, and the 3D method took a block as input. UNet [17] was more commonly used in the 2D method. However, 3D-UNet [18] replaced 2D convolution in UNet with 3D convolution. In this study, to propose 2D-3D CNN and achieve better segmentation effect of pancreas, the semantic information of single slice extracted by the 2D method and contextual semantic information extracted by the 3D method were combined. Data preprocessing was as the following: the data setting of the study was 136 CT images. 36 were used for training, and 100 were used for testing. The scanning resolution was 512 × 512 pixels, and the layer thickness was 1.2 ~ 2.5 mm. The data set was preprocessed, and the processing process was as the following:

As the original abdominal CT images had different ranges of Hounsfield unit (HU) in different tissues, the range of HU in the pancreas was generally 30~ 35. The study calculated the extent of the pancreas on account of the Hu-Pixel conversion equation. The equation was as the following:

(1) $$\begin{array}{c} \text{HU}=\text{Pixel}*\text{ScaleFactor}+\text{Bias}. \end{array}$$

In Equation (1), Pixel was pixel value, ScaleFactor was scaling ratio, and Bias was Bias. Then, it was suggested to truncate the data according to the calculated pancreatic window. The truncated data were selected to standardize the spread. The equation was as the following:

(2) $$\begin{array}{c} Y=\frac{\left(M-m^{\min}\right)}{\left(m^{\max}-m^{\min}\right)}. \end{array}$$

Given the relatively fixed location of the pancreas, the study placed pancreatic location statistics first. According to the statistical location data, the pancreas was segmented and cropped to reduce the original image from 512 × 512 pixels to 256 × 256 pixels. The image was then cropped to 128 × 128 pixels using quadratic linear difference.

Pancreas was segmented by 2D-3D CNN. 2D-3D CNN used in this study was divided into 2D single slice semantic part and 3D context semantic part. 2D CNN was introduced into residual neural network (ResNet). Encoder parameters were set as 64, 128, 256, 512, and 1,024. The number of residual units in each residual group was set as 1, 1, 1, and 1. The convolutional layer and deconvolution layer with step size of 2 were used for up-down sampling. 3D part introduced ResNet18-3D velocity net network. Decoder parameters were set as 32, 64, 128, and 256. The number of residual units of each residual group was set as 2, 2, 2, and 2. The convolutional layer and deconvolution layer with step size of 2 were used for up-down sampling.

The segmentation process was shown in Figure 1:

### 2.5. Model Training

CT image data of pancreatic cancer were obtained from CT images. 36 of them were selected for model training, and 100 were selected for model testing. Due to large differences between 2D and 3D image features, the model might fail to converge, thus affecting the segmentation result, which should be taken into account. Therefore, the 2D model was firstly trained separately in this study. After 2D network parameters were set, the 3D model was trained. Finally, 2D and 3D models were trained simultaneously.

### 2.6. Observation Indicators

The serum levels of CA-50, CA-199, and CA-242 were compared between two groups. The diagnostic efficacy indexes of the three tumor markers were analyzed, including sensitivity, specificity, accuracy, positive predictive value, negative predictive value, and true value, which were shown in the following equations:

(3) $$\begin{array}{c} \text{Accuracy}=\frac{\text{TP}+\text{TN}}{\text{TP}+\text{TN}+\text{FP}+\text{FN}}, \end{array}$$

(4) $$\begin{array}{c} \text{Sensitivity}=\frac{\text{TP}}{\text{TP}+\text{FN}}, \end{array}$$

(5) $$\begin{array}{c} \text{Specificity}=\frac{\text{TN}}{\text{FP}+\text{TN}}. \end{array}$$

In Equations (3)–(5), TP represented true positive of test results. FN was false negative. FP was false positive. TN was true negative. In this study, the effect of CT image segmentation was evaluated by using Dice coefficient. *Z* was the result of manual segmentation by experts. *D* was the segmentation result of the algorithm designed in this study, which was shown in Equation (6):

(6) $$\begin{array}{c} \text{Dice}=\frac{2\left|\text{Z}⋂\text{D}\right|}{\left|\text{Z}\right|+\left|\text{D}\right|}. \end{array}$$

### 2.7. Statistical Analyses

SPSS 21.0 statistical software was used for data processing and analyses. *t*-test was used for intergroup comparison. Diagnostic efficacy such as sensitivity, specificity, and accuracy was used as counting data and expressed as rates. Chi-square test was used for intergroup comparison, and *P* < 0.05 indicated statistically significant differences.

## 3. Results

### 3.1. Algorithm Performance Evaluation

The study compared the training results of 2D, 3D, and 2D-3D in 36 pancreatic maps, as shown in Figure 2. The maximum, minimum, and average values of 2D training results were 89.75%, 62.37%, and 82.32%, respectively. The maximum value, minimum value, and average value of 3D training results were 89.86%, 56.42%, and 81.76%, respectively. The maximum, minimum, and average values of 2D-3D training results were 91.32%, 68.21%, and 84.27%, respectively. Thus, the 2D-3D method was more stable and reliable.

The FCN [19] algorithm was also introduced in the study. FCN, UNet, and 2D-3D algorithm were compared in the test results of 100 pancreatic CT images, as shown in Figure 3. The maximum value, minimum value, and average value of the UNet algorithm were 88.12%, 64.32%, and 80.62%, respectively. The maximum value, minimum value, and average value of the FCN algorithm were 87.63%, 63.79%, and 79.26%, respectively. The maximum value, minimum value, and average value of the 2D-3D algorithm were 90.75%, 67.14%, and 84.32%, respectively. The segmentation effect of the 2D-3D algorithm was better than the other two algorithms, and the differences were statistically significant (*P* < 0.05).

Figure 4 was the segmentation effect diagram of the 2D-3D convolution neural algorithm.

### 3.2. Comparison of CT Signs of Patients

CT signs of patients in two groups were counted, including included lesions, peripheral blood vessels, and pancreatic duct, which were shown in Figure 5. In Figure 5(a), the lesions of two groups were compared. In the experimental group, the proportion of unclear lesion edge, cystic lesion, calcification in lesion, and uneven enhancement was 88.32%, 23.17%, 3.17%, and 53.68%, respectively. The proportion of cystic lesion and calcification in lesion was higher than that in the control group, but there was no statistical significance (*P* > 0.05). In Figure 5(b), conditions of peripheral blood vessels and pancreatic ducts were compared between two groups. The proportion of pancreatic duct dilation, pancreatic duct penetration sign, vascular involvement, and pancreatic portal hypertension in the experimental group was 63.16%, 22.12%, 58.02%, and 43.15%, respectively. The proportion of pancreatic duct penetration was lower than that in the control group, with statistical significance (*P* < 0.05).

### 3.3. Comparison of CT Values of Patients

CT value was generally expressed as HU. In this study, CT values of plain scan, arterial phase, portal vein phase, and delayed phase were compared between two groups, and the results were shown in Figure 6. CT values of plain scan, arterial phase, portal vein phase, and delayed phase in the experimental group were 36.87, 50.21, 72.18, and 78.93, respectively. CT values of plain scan, arterial phase, portal vein phase, and delayed phase in the experimental group were 35.43, 61.17, 74.49, and 80.21, respectively. CT value of arterial phase in the experimental group was significantly lower than that in the control group, and the differences were statistically significant (*P* < 0.05).

### 3.4. Serum Tumor Marker Level Statistics of Patients

Serum tumor marker levels of two groups were shown in Figure 7. CA-50, CA-199, and CA-242 in the experimental group were 141.72 U/mL, 1548.24 U/mL, and 83.65 U/mL, respectively. CA-50, CA-199, and CA-242 in the control group were 29.18 U/mL, 74.83 U/mL, and 12.53 U/mL, respectively, which were significantly lower than the experimental group, and the differences were statistically significant (*P* < 0.05).

### 3.5. Analyses of Diagnostic Performance of Serum Tumor Markers and Combined Detection of Serum Tumor Markers

This study analyzed the diagnostic value of tumor markers CA-50, CA-199, CA-242, and their combined detection for pancreatic cancer, as shown in Figure 8. The sensitivity, specificity, positive predictive value, negative predictive value, and authenticity of combined detection of serum tumor markers were 89.31%, 92.31%, 84.75%, 87.79%, and 86.32%, respectively. Its sensitivity, specificity, positive predictive value, and authenticity were higher than those of CA-50, CA-199, and CA-242, and the differences were statistically significant (*P* < 0.05).

### 3.6. Diagnostic Performance Analyses of CT and CT Combined with Serum Tumor Markers

As could be shown from the test results in 3.5 above, the combined detection of serum tumor markers had better diagnostic performance than the single detection of serum tumor markers. Therefore, this study analyzed the diagnostic performance of CT and CT combined with tumor marker (CT-STUM) for pancreatic cancer, and the results were shown in Figure 9. The sensitivity, specificity, positive predictive value, negative predictive value, and authenticity of CT-STUM were 94.57%, 93.25%, 84.57%, 90.34%, and 87.63%, respectively, which were higher than those of CT, and the differences were statistically significant (*P* < 0.05).

### 3.7. Patient Images

Figure 10 shows the image data of plain CT scan, CT arterial enhancement, venous phase, and delayed phase of an 88-year-old male patient. The patient's pancreas was locally enlarged with mass formation, and the boundary of the pancreas was not clear. The density increase was not obvious when the plain mass was presented with isodensity enhanced scan.

## 4. Discussion

The degree of malignancy of pancreatic cancer is relatively high, and its location is hidden. All diagnostic methods in clinical practice have certain limitations, which greatly affect the prognosis of patients [20]. Serum tumor markers CA-50, CA-199, and CA-242 play a role in diagnoses of pancreatic cancer. However, there are certain false positives in the test method, which is consistent with the test results of this study [21]. The high resolution of CT diagnoses has certain diagnostic value for pancreas with special location. However, CT detection results can only show the appearance of pancreas and are subject to large factors of imaging results and subjective judgments of clinicians, which may lead to misdiagnoses and missed diagnosis [22–24]. Therefore, this study proposed a 2D-3D CNN segmentation algorithm on account of the intelligent algorithm and used it to the feature analyses of pancreatic cancer CT images. Combined with serum tumor markers CA-50, CA-199, and CA-242, the diagnostic value of the combined detection method for pancreatic cancer was comprehensively analyzed.

Dice coefficient results of 2D, 3D, and 2D-3D CNN training were compared. The maximum value, minimum value, and average value of 2D-3D training results were 91.32%, 68.21%, and 84.27%, respectively, which were higher than those of 2D and 3D CNNs, proving that the 2D-3D CNN segmentation algorithm had good stability. In order to further analyze the segmentation performance of the algorithm, FCN and UNet algorithms were also introduced. The test results showed that the maximum and average Dice coefficient of the 2D-3D CNN segmentation algorithm was 90.75% and 84.32%, and both were higher than the other two algorithms. It showed that the 2D-3D CNN segmentation algorithm proposed in this study had the best effect on CT image processing and has clinical promotion value. Such results are similar to the research results of Gupta et al. [25]. They proposed a consistent CT image reconstruction algorithm based on CNN and compared it with a regularization reconstruction algorithm based on total variation and a dictionary learning reconstruction algorithm, and it was found that the CNN consistent image reconstruction algorithm has made significant progress compared with the traditional algorithm. Subsequently, the designed algorithm was used to the CT imaging evaluation of pancreatic cancer, and the CT signs of two groups were compared. The proportions of pancreatic duct dilatation, pancreatic duct crossing sign, vascular involvement, and pancreatic portal hypertension in the experimental group were 63.16%, 22.12%, 58.02%, and 43.15%, respectively. The proportion of pancreatic duct penetration was lower than that of control group, the rest was higher than that of control group, and the differences were statistically significant (*P* < 0.05). It further showed that CT images based on the 2D-3D CNN segmentation algorithm can effectively display the lesions of pancreatic cancer patients.

The study compared serum tumor marker levels between two groups. CA-50, CA-199, and CA-242 in the experimental group were 141.72 U/mL, 1548.24 U/mL, and 83.65 U/mL, respectively, which were higher than those in control group, and the differences were statistically significant (*P* < 0.05). On account of this, the study compared the diagnostic value of three serum tumor markers for pancreatic cancer. The sensitivity, specificity, positive predictive value, negative predictive value, and authenticity of combined detection of serum tumor markers were 89.31%, 92.31%, 84.75%, 87.79%, and 86.32%, respectively. Its sensitivity, specificity, positive predictive value, and authenticity were higher than those of CA-50, CA-199 and CA-242, and the differences were statistically significant (*P* < 0.05). Finally, the diagnostic value of CT and CT combined with serum tumor markers in pancreas was compared between two groups. The results showed that the sensitivity, specificity, positive predictive value, negative predictive value, and authenticity of CT-STUM were 94.57%, 93.25%, 84.57%, 90.34%, and 87.63%, respectively, which were higher than those of CT, and the difference was statistically significant (*P* < 0.05). This study result was similar to Jung et al. [26].

## 5. Conclusion

In this study, 68 hospitalized patients with pancreatic cancer were included in the experimental group, and 68 hospitalized patients with chronic pancreatitis were undertaken as the control group, all underwent CT imaging. In addition, a 2D-3D CNN segmentation algorithm was proposed for CT image enhancement processing, and the diagnostic efficiency of CT combined with serum tumor markers based on intelligent algorithms was analyzed for pancreatic cancer. The result revealed that compared with FCN and UNet, the image segmentation algorithm designed in this study had better algorithm stability and image segmentation performance. CT combined with tumor marker detection had higher sensitivity and specificity for diagnoses of pancreatic cancer, and its diagnostic effect was the best. However, the study lacked the diagnostic performance analyses of other tumor markers for pancreatic cancer except CA-50, CA-199, and CA-242. In the following research, the comprehensive segmentation performance of the 2D-3D CNN algorithm needs to be further verified. Overall, the results of this study provided reliable data support for clinical diagnoses and prognosis of patients with pancreatic cancer.

## Figures and Tables

**Figure 1:** 2D-3D CNN segmentation process.

**Figure 2:** 2D, 3D, and 2D-3D training results.

**Figure 3:** Test results of the three algorithms. Notes: ∗ represented statistically significant differences compared with the 2D-3D algorithm (*P* < 0.05).

**Figure 4:** 2D-3D convolutional neural algorithm segmentation effect diagram. Notes: (a) was the abdominal CT image, (b) was the corresponding label, and (c) was the segmentation result.

**Figure 5:** Comparison of CT signs of patients. Notes: (a) showed the lesions. (b) showed pancreatic duct and other conditions. ∗ showed statistically significant differences compared with the experimental group (*P* < 0.05).

**Figure 6:** Comparison of CT values of patients. Notes: ∗ indicated statistically significant differences compared with experimental group (*P* < 0.05).

**Figure 7:** Serum tumor marker level statistics of patients. Notes: ∗ indicated statistically significant differences compared with the experimental group (*P* < 0.05).

**Figure 8:** Diagnostic performance analyses of serum tumor markers. Notes: (a) was CA-50, (b) was CA-199, (c) was CA-242, and (d) was the combined detection. Photovoltaic was the predicted value.

**Figure 9:** Diagnostic performance analyses of CT and CT combined with serum tumor markers. Note: ∗ indicated statistically significant differences compared with CT-STUM (*P* < 0.05).

**Figure 10:** CT imaging data of the patient. Notes: (a) was the plain CT, (b) was the CT arterial enhancement, (c) was the venous stage, and (d) was the delay period.

## Data Availability

The data used to support the findings of this study are available from the corresponding author upon request.
